The article "Autophagy Is Required for Hepatic Differentiation of Hepatic Progenitor Cells via Wnt Signaling Pathway" was published in 2021. Journal: Biomed Res Int.

# Autophagy Is Required for Hepatic Differentiation of Hepatic Progenitor Cells via Wnt Signaling Pathway

**DOI:** 10.1155/2021/6627506

**Published:** 2021-04-08

**Authors:** Jianxing Zeng, Yingying Jing, Qionglan Wu, Jinhua Zeng, Lixin Wei, Jingfeng Liu

**Affiliations:** ^1^Department of Hepatic Surgery, Mengchao Hepatobiliary Hospital of Fujian Medical University, Fuzhou 350025, China; ^2^The First Affiliated Hospital of Fujian Medical University, Fuzhou 350005, China; ^3^Fujian Provincial Medical Center of Hepatobiliary, Fuzhou 350025, China; ^4^Tumor Immunology and Gene Therapy Center, Eastern Hepatobiliary Surgery Hospital, The Second Military Medical University, Shanghai 200438, China; ^5^Department of Pathology, Mengchao Hepatobiliary Hospital of Fujian Medical University, Fuzhou 350025, China

## Abstract

The molecular mechanisms regulating differentiation of hepatic progenitor cells (HPCs), which play pivotal roles in liver regeneration and development, remain obscure. Autophagy and Wnt signaling pathways regulate the development and differentiation of stem cells in various organs. However, the roles of autophagy and Wnt signaling pathways in hepatic differentiation of HPCs are not well understood. Here, we describe the effects of autophagy and Wnt signaling pathways during hepatic differentiation of HPCs. We used a well-established rat hepatic progenitor cell line called WB-F344, which was treated with differentiation medium to promote differentiation of WB-F344 cells along the hepatic phenotype. Firstly, autophagy was highly activated in HPCs and gradually decreased during hepatic differentiation of HPCs. Induction of autophagy by rapamycin or starvation suppressed hepatic differentiation of HPCs. Secondly, Wnt3a signaling pathway was downregulated, and Wnt5a signaling pathway was upregulated in hepatic differentiation of HPCs. At last, Wnt3a signaling pathway was enhanced, and Wnt5a signaling pathway was inhibited by activation of autophagy during hepatic differentiation of HPCs. In summary, these results demonstrate that autophagy regulates hepatic differentiation of hepatic progenitor cells through Wnt signaling pathway.

## 1. Introduction

Chronic liver disease is a common clinical liver disease with high morbidity and mortality worldwide [1]. The only cure for end-stage chronic liver disease is liver transplantation; however, donor organ availability cannot meet demand [2]. For this reason, other alternative treatment strategies like controlling regeneration in chronic liver disease become adapted and developed [3]. The liver regeneration usually comes from hepatic progenitor cells (HPCs) [4]. HPCs are multipotent stem cells resided within a central component of the ductular reaction, which differentiate into hepatocyte or cholangiocyte in an activated niche to regenerate the damaged liver [5, 6]. The differentiation of HPCs has been reported to be regulated by various signaling pathways, including autophagy, Notch, Wnt, bone morphogenetic protein (BMP), hepatocyte growth factor (HGF), and fibroblast growth factor (FGF) signaling pathways [7, 8]. Therefore, the mechanism regulating the differentiation of HPCs is complex and unclear; it is necessary to understand the mechanisms regulating the differentiation of HPCs into functional hepatocytes.

The article "Autophagy Is Required for Hepatic Differentiation of Hepatic Progenitor Cells via Wnt Signaling Pathway" was published in 2021. Journal: Biomed Res Int.

Wnt signaling pathway plays a crucial role in the differentiation, proliferation, and self-renewal of stem cells in various organs [9, 10]. Traditionally, the Wnt signaling pathway is classified into two categories: the canonical Wnt (or *β*-catenin-dependent) and noncanonical Wnt (or *β*-catenin-independent) signaling pathways [11]. The canonical and noncanonical signaling pathways form intersecting signaling networks that coordinately regulate complex processes, such as embryonic development, stem cell maintenance and differentiation, and tissue homeostasis [12–15]. A recent study has demonstrated that noncanonical Wnt signaling pathway plays an important role in modulating canonical Wnt-regulated stemness, proliferation, and differentiation of HPCs [16].

Autophagy is an evolutionarily conserved ubiquitous process in eukaryotic cells [17]. Autophagy has been characterized as an essential process associated with cellular homeostasis [18]. Under stress or starvation conditions, autophagy-related protein P62 delivers unnecessary and damaged biomacromolecules and organelles in the cytoplasm to lysosomes for degradation via double-membrane autophagosomes, thus promoting cell survival and growth [19]. Recent studies have shown autophagy plays a crucial part in the self-renewal and differentiation of stem cells [20–23]. We previously reported that autophagy regulated biliary differentiation of HPCs through Notch1 signaling pathway [24]. Autophagy also regulates Wnt signaling pathway in cell development and differentiation [25–27]. However, whether autophagy regulates Wnt signaling pathway in hepatic differentiation is not well understood.

In this study, we investigated the roles of autophagy and Wnt signaling pathways during the hepatic differentiation process of HPCs. We found that autophagy was highly activated in HPCs and gradually decreased during hepatic differentiation of HPCs. Induction of autophagy by rapamycin or starvation suppressed hepatic differentiation of HPCs. Further study reported that Wnt3a signaling pathway was downregulated, and Wnt5a signaling pathway was upregulated in hepatic differentiation of HPCs. Wnt3a signaling pathway was enhanced, and Wnt5a signaling pathway was inhibited by activation of autophagy during hepatic differentiation of HPCs. These results demonstrate that autophagy regulates hepatic differentiation of hepatic progenitor cells through Wnt signaling pathway.

The article "Autophagy Is Required for Hepatic Differentiation of Hepatic Progenitor Cells via Wnt Signaling Pathway" was published in 2021. Journal: Biomed Res Int.

## 2. Materials and Methods

### 2.1. Reagents

The P62 (Cell Signaling Technology, Danvers, Massachusetts, USA), LC3A/B (Cell Signaling Technology, Danvers, Massachusetts, USA), Alb (Santa Cruz Biotechnology, Inc, Dallas, Texas, USA), Aldob (Santa Cruz Biotechnology, Inc, Dallas, Texas, USA), Wnt3a (Abcam, Cambridge, UK), *β*-catenin (Abcam, Cambridge, UK), Sox9 (Merck KGaA, Darmstadt, Germany), Wnt5a (Abcam, Cambridge, UK), CaMKII*α* (Cell Signaling Technology, Danvers, Massachusetts, USA), Phospho-CaMKII*α* (Thr286) (Cell Signaling Technology, Danvers, Massachusetts, USA), and Actin (Bioworld Technology, Bloomington, USA) antibodies were used for Western blotting staining. HGF (315–23) and EGF (400–25) were obtained from Peprotech. OSM (495-MO) was purchased from R&D Systems. ITS-X (51500–056) was obtained from Lifetech. 2-Mercaptoethanol (21985023) was purchased from Thermo Fisher Scientific. VitC (A4403) and nicotinamide (N0636) were purchased from Sigma-Aldrich. Dexamethasone and gentamicin were purchased from Mengchao Hepatobiliary Hospital of Fujian Medical University.

### 2.2. Cell Culture and Treatments

WB-F344 cells were purchased from the Chinese Academy of Sciences, Shanghai. WB-F344 cells were cultured in Dulbecco's Modified Eagle Medium (DMEM) supplemented with 4.5 g/L glucose and 10% foetal bovine serum (FBS) at 37°C with 5% CO_2_. WB-F344 cells were cultured with DMEM supplemented with 4.5 g/L glucose, 10% FBS, 0.1 mmol/L 2-mercaptoethanol, 1x ITS-X, 10 ng/mL HGF, 20 ng/mL EGF, 20 ng/mL OSM, 0.5 mmol/L VitC, 50 mg/mL gentamicin, 10 mmol/L nicotinamide, and 10^−6^ mol/L dexamethasone for 4 days for hepatocyte differentiation. We examined the effects of two autophagy stimuli, mTOR inhibitor rapamycin, and cell starvation, on hepatic differentiation of WB-F344 cells. WB-F344 cells were treated with hepatic differentiation medium for 2 days and cocultured rapamycin 200 nM for 24 h or serum-free medium for starve 24 h.

### 2.3. Western Blotting Analysis

Treated cells were washed with phosphate buffer saline (PBS) and lysed with RIPA buffer containing PMSF at a ratio of 100 : 1 to obtain total protein for Western blot analysis. Proteins were separated by electrophoresis on 10–12% SDS-polyacrylamide gels, transferred to polyvinylidene fluoride membrane, and incubated with corresponding primary antibodies overnight at 4°C. Following incubated with secondary antibody 1 h at room temperature. Immunoblots were developed using the BeyoECL (Beyotime) and Tanon 5200 system, and the blot was scanned and densitometric analysis with the Image J software. The primary antibodies are used in our experiment including P62 (1 : 1000), LC3A/B (1 : 1000), Alb (1 : 1000), Aldob (1 : 1000), Wnt3a (1 : 1000), *β*-catenin (1 : 5000), Sox9 (1 : 1000), Wnt5a (1 : 1000), CaMKII*α* (1 : 1000), Phospho-CaMKII*α* (Thr286) (1 : 1000), and Actin (1 : 5000).

The article "Autophagy Is Required for Hepatic Differentiation of Hepatic Progenitor Cells via Wnt Signaling Pathway" was published in 2021. Journal: Biomed Res Int.

### 2.4. Cell Proliferation Assay

Cell proliferation was measured by Cell Counting Kit-8 (CCK8, Dojindo, Japan) assay according to the manufacturer's instructions. Experiments for CCK8 were performed in 96-well plates. Cells were seeded at a density of 1 × 10^4^ cells/mL. 20 *μ*L CCK-8 solution was added into each well (containing 200 *μ*L medium) and further cultured for 2 h at 37°C. The absorbance of each group at 450 nm was detected using an absorbance microplate reader.

### 2.5. Real-Time Polymerase Chain Reaction (RT-PCR)

Total RNA from different groups of cells was extracted using TRIZOL reagent (Invitrogen, USA) according to the manufacturer's protocol. RT-PCR was performed using SYBR Green PCR Kit. The relative quantities of mRNAs were obtained by using the comparative Ct method and were normalized with glyceraldehydes-3-phosphate dehydrogenase (GAPDH). The primers were presented in Table 1.

### 2.6. Electron Microscopic Analysis

Cells were fixed in 2.5% glutaraldehyde in PBS for 2 h at room temperature, then fixed in 1% osmium tetroxide in water for 1 h, dehydrated in an ascending series of ethanol, and at last embedded in Araldite (Basel, Switzerland). After solidified, 50 nm sections were cut on LKB-I ultramicrotome and picked up on copper grids, poststained with uranyl acetate and lead citrate, and observed in a Philips CM-120 TEM.

### 2.7. Statistical Analysis

All of the experiments were repeated at least 3 times. Data was expressed as mean ± standard deviation (SD). Statistical analysis of the data was done by using GraphPad Prism 6. The student's *t*-test was used to compare between mean values of the two groups. *P* < 0.05 was considered statistically significant.

## 3. Results

### 3.1. Autophagy Was Highly Activated in HPCs and Gradually Decreased during Hepatic Differentiation of HPCs

To investigate whether autophagy was involved in hepatic differentiation of HPCs, we used a well-established rat hepatic progenitor cell line called WB-F344, which was treated with differentiation medium to promote differentiation of WB-F344 cells along the hepatic phenotype. First, the morphology of WB-F344 cells was notably changed (Figure 1(a)). Second, the hepatic lineage makers Alb and Aldob were also significantly increased (Figures 1(b) and 1(c)). Third, the proliferation ability of WB-F344 cells with differentiation medium for 4 days was significantly lower than that of normal medium (Figure 1(d)), indicating that WB-F344 cells could differentiate into hepatocytes in differentiation medium.

The article "Autophagy Is Required for Hepatic Differentiation of Hepatic Progenitor Cells via Wnt Signaling Pathway" was published in 2021. Journal: Biomed Res Int.

Next, we detected the level of autophagy (LC3-II/LC3-I and P62) during the progression of hepatic differentiation. We observed that the level of LC3-II/LC3-I was highly activated in WB-F344 cells; when treated with differentiation medium, LC3-II/LC3-I level was gradually decreased (Figure 1(e)). On the contrary, the P62 level was increased (Figure 1(e)). The quantitation of LC3-II/LC3-I was also decreased (Figure 1(f)). To observe the formation of autophagic vacuoles intuitively, the electron microscopy was employed. Without differentiation medium induction, autophagic vacuoles were easy to detect in WB-F344 cells. Oppositely, autophagic vacuoles were few in WB-F344 cells treated with differentiation medium for 4 days (Figure 1(g)). These results showed that autophagy was highly activated in HPCs and gradually decreased during the progression of hepatic differentiation.

### 3.2. Induction of Autophagy Suppressed Hepatic Differentiation of HPCs

To further investigate the effect of autophagy on hepatic differentiation of HPCs, we examined the effects of two autophagy stimuli, mTOR inhibitor rapamycin and nutrient deprivation medium, on hepatic differentiation of WB-F344 cells. WB-F344 cells were treated with differentiation medium for 2 days and cocultured DMSO, rapamycin, or starvation for 24 h. Western blot analysis indicated that LC3-II/LC3-I level was increased, and P62 level was decreased by rapamycin (Figure 2(a)) or starvation (Figure 2(d)). Rapamycin decreased the expression of Alb and Aldob relative to DMSO (Figures 2(b) and 2(c)). Starvation also attenuated the expression of Alb and Aldob relative to DMSO (Figures 2(e) and 2(f)). These results indicated that activation of autophagy suppressed hepatic differentiation of HPCs.

### 3.3. Wnt Signaling Pathway Was Involved during Hepatic Differentiation of HPCs

We have demonstrated that activation of autophagy suppressed hepatic differentiation of HPCs. Next, we explored how autophagy influenced hepatic differentiation. We firstly investigated whether Wnt signaling pathway took part in hepatic differentiation of HPCs. After exposing to differentiation medium for 4 days, the expression of Wnt3a was decreased, and Wnt5a was elevated; Wnt1, Wnt4, and Wnt 9a were not change (Figure 3(a)). Meanwhile, the expressions of *β*-catenin (central role of Wnt3a signaling pathway), Sox9, and Axin2 (target transcripts of Wnt3a signaling pathway) were downregulated during hepatic differentiation of WB-F344 cells (Figures 3(b) and 3(c)). Western blot analysis revealed that the levels of Wnt5a and phosphorylated CaMKII*α* (P-CaMKII*α*) were increased (Figure 3(d)). These data demonstrated that Wnt3a signaling pathway was downregulated, and Wnt5a signaling pathway was upregulated in hepatic differentiation of HPCs.

The article "Autophagy Is Required for Hepatic Differentiation of Hepatic Progenitor Cells via Wnt Signaling Pathway" was published in 2021. Journal: Biomed Res Int.

### 3.4. Autophagy Regulated Wnt Signaling Pathway during Hepatic Differentiation of HPCs

To further investigate whether Wnt signaling pathway could be regulated by autophagy during hepatic differentiation of HPCs. We also examined the effect of two autophagy stimuli, mTOR inhibitor rapamycin and starvation, on hepatic differentiation of WB-F344 cells. The expression of Wnt3a, *β*-catenin, Sox9, and Axin2 were significantly higher in cultured cells supplemented with rapamycin relative to DMSO (Figures 4(a)–4(c)). The expression of Wnt5a and P-CaMKII*α* were significantly downregulated in cultured cells supplemented with rapamycin relative to DMSO (Figures 4(a) and 4(d)). Starvation also promoted the expression of Wnt3a, *β*-catenin, Sox9, and Axin2 (Figures 4(e)–4(g)) and attenuates the expression of Wnt5a and P-CaMKII*α* relative to DMSO (Figures 4(e) and 4(h)), indicating that Wnt3a signaling pathway was enhanced and Wnt5a signaling pathway was inhibited by activation of autophagy during hepatic differentiation of HPCs.

## 4. Discussion

Hepatocytes have sufficient regenerative capacity [28]. This regenerative ability is enhanced in chronic liver disease with the ductular reactions (DR) [29]. Within the DR are cells that express both bile duct cell and hepatocyte features [30, 31]. It is thought that these cells can be hepatic progenitor cells (HPCs) that differentiate into both hepatocytes and cholangiocytes [5, 6]. It has been reported that the differentiation of HPCs is regulated by a variety of signaling pathways, including autophagy, Notch, Wnt, BMP, HGF, and FGF signaling pathways [7, 8]. In this study, we demonstrated that autophagy and Wnt signaling pathways regulated hepatic differentiation of HPCs.

Wnt signaling pathway plays an essential role in liver development [13, 32]. Wnt1, Wnt2, Wnt3, Wnt3a, Wnt7b, Wnt8a, and Wnt8b have shown a preferential ability to signal through *β*-catenin [14]. Similarly, Wnt4, Wnt5a, Wnt9a, Wnt10a, and Wnt11 were reported to emit signals through different intracellular signaling mechanisms, including Ca^2+^-mediated pathways or the c-Jun N-terminal kinase cascade [15]. Generally, the canonical Wnts that signal through *β*-catenin associate to cell proliferation, while the noncanonical Wnts seem to promote differentiation and oppose proliferation and cellular multipotency [33]. Specifically, Wnt5a is shown to promote differentiation in a variety of tissues while opposing the proliferative effects of canonical Wnts, including Wnt1 and Wnt3a [16, 34]. Our data showed that the stemness and proliferation of hepatic progenitor cells were regulated by Wnt3a/*β*-catenin pathway. On the other hand, Wnt5a/Ca^2+^-mediated pathway was shown to promote differentiation of hepatic progenitor cells.

The article "Autophagy Is Required for Hepatic Differentiation of Hepatic Progenitor Cells via Wnt Signaling Pathway" was published in 2021. Journal: Biomed Res Int.

An increasing number of studies have shown that autophagy plays a vital role in stem cell maintenance and differentiation [20, 23, 35]. It has been reported that autophagy regulates stemness and self-renewal of HPCs [36]. We previously reported that autophagy regulated biliary differentiation of HPCs through Notch1 signaling pathway [24]. In this study, we found that high autophagic activity is observed in HPCs and decreased in the process of hepatic differentiation. Activation of autophagy by rapamycin or starvation suppressed hepatic differentiation of HPCs.

Autophagy is also reported to be related to Wnt signaling pathway in different cell models. Autophagy negatively regulates Wnt signaling by promoting Disheveled (Dvl) degradation in the late stages of colon cancer development [25]. *β*-Catenin suppresses autophagosome formation and directly repressed the autophagy adaptor P62 expression [26]. Autophagy stimulates the proliferation of porcine pancreatic stem cells, which is regulated by the canonical Wnt signaling pathway [37]. Autophagy eliminates cytoplasmic *β*-catenin to promote cardiac differentiation [27]. However, whether autophagy regulates Wnt signaling pathway in hepatic differentiation is not clear. In our study, we found that autophagy was decreased, and canonical Wnt pathway (Wnt3a/*β*-catenin) was suppressed, and noncanonical Wnt pathway (Wnt5a/Ca^2+^) was enhanced during hepatic differentiation of HPCs; activation of autophagy was enhanced Wnt3a/*β*-catenin signaling pathway and impeded hepatic differentiation. *β*-Catenin plays a key role in the transduction of Wnt pathway [14]. Therefore, autophagy may regulate *β*-catenin during hepatic differentiation of HPCs. Although the study of the mechanism underlying hepatic differentiation of HPCs is not sufficiently explained, the results will be helpful to further understand the mechanism of hepatic differentiation of HPCs.

## 5. Conclusion

The present results describe a direct link between autophagy and Wnt signaling pathways, both of which regulated hepatic differentiation. Firstly, autophagy was highly activated in HPCs and gradually decreased during hepatic differentiation of HPCs. Induction of autophagy by rapamycin or starvation suppressed hepatic differentiation of HPCs. Secondly, Wnt3a signaling pathway was downregulated, and Wnt5a signaling pathway was upregulated in hepatic differentiation of HPCs. At last, Wnt3a signaling pathway was enhanced, and Wnt5a signaling pathway was inhibited by activation of autophagy during hepatic differentiation of HPCs. These results demonstrate that autophagy regulates hepatic differentiation of hepatic progenitor cells through Wnt signaling pathway.

The article "Autophagy Is Required for Hepatic Differentiation of Hepatic Progenitor Cells via Wnt Signaling Pathway" was published in 2021. Journal: Biomed Res Int.

## Figures and Tables

**Figure 1:** Autophagy was highly activated in HPCs and gradually decreased during hepatic differentiation of HPCs. (a) The morphology of WB-F344 cells cultured in normal medium (left panel, Ctrl, control) or treated with hepatic differentiation medium (HGF) for 4 days (right panel, HGF) (scale bars = 20 *μ*m, Inset: 2x magnification). (b) RT-PCR analyzing expression of hepatic lineage markers (Alb and Aldob) in WB-F344 cells treated with hepatic differentiation medium (HGF) for 4 days. (c) Western blot showing expression of hepatic lineage markers (Alb and Aldob) in WB-F344 cells treated with hepatic differentiation medium (HGF) for 4 days. (d) The proliferation ability of WB-F344 cells cultured in normal medium (Ctrl) or treated with hepatic differentiation medium (HGF) for 4 days. (e) Western blot showing autophagy (LC3-II/LC3-I and P62) in WB-F344 cells treated with hepatic differentiation medium (HGF) for 4 days. (f) Densitometric analysis of LC3-II relative to LC3-I normalized to time 0 d (0 d vs. 1 d-4 d). (g) Autophagic vacuoles (arrowheads) were observed at WB-F344 cells cultured in normal media (Ctrl) or treated with differentiation medium (HGF) for 4 days under an electron microscope (scale bars = 1 *μ*m). Data represent mean ± SD; ^∗^*P* < 0.05; ^∗∗^*P* < 0.01. *n* = 3.

**Figure 2:** Induction of autophagy suppressed hepatic differentiation of HPCs. (a) Western blot showing the level of LC3-II/LC3-I and P62 in WB-F344 cells treated with differentiation medium (HGF) for 2 days and coculture DMSO or rapamycin (200 nM; Rapa) for 24 h. (b) RT-PCR analyzing the expression of hepatic lineage markers (Alb and Aldob) in WB-F344 cells treated with differentiation medium (HGF) for 2 days and coculture DMSO or rapamycin (200 nM; Rapa) for 24 h. (c) Western blot showing the expression of hepatic lineage markers (Alb and Aldob) in WB-F344 cells treated with differentiation medium (HGF) for 2 days and coculture DMSO or rapamycin (200 nM; Rapa) for 24 h. (d) Western blot showing the level of LC3-II/LC3-I and P62 in WB-F344 cells treated with differentiation medium (HGF) for 2 days and coculture DMSO or starvation (serum-free medium; Starve) for 24 h. (e) RT-PCR analyzing the expression of hepatic lineage markers (Alb and Aldob) in WB-F344 treated with differentiation medium (HGF) for 2 days and coculture DMSO or starvation (serum-free medium; Starve) for 24 h. (f) Western blot showing the expression of hepatic lineage markers (Alb and Aldob) in WB-F344 treated with differentiation medium (HGF) for 2 days and coculture DMSO or starvation (serum-free medium; Starve) for 24 h. Data represent mean ± SD; ^∗^*P* < 0.05. *n* = 3.

The article "Autophagy Is Required for Hepatic Differentiation of Hepatic Progenitor Cells via Wnt Signaling Pathway" was published in 2021. Journal: Biomed Res Int.

**Figure 3:** Wnt signaling pathway was involved during hepatic differentiation of HPCs. (a) RT-PCR analyzing the mRNA expression of Wnt1, Wnt3a, Wnt4, Wnt5a, and Wnt9a in WB-F344 cells treated with hepatic differentiation medium (HGF) for 4 days. (b) RT-PCR analyzing the mRNA expression of *β*-catenin, Sox9, and Axin2 in WB-F344 cells treated with hepatic differentiation medium (HGF) for 4 days. (c) Western blot showing the level of Wnt5a, P-CaMKII*α*, and CaMKII*α* in WB-F344 cells treated with hepatic differentiation medium (HGF) for 4 days. (d) Western blot showing the level of Wnt3a, *β*-catenin, and Sox9 in WB-F344 cells treated with hepatic differentiation medium (HGF) for 4 days. Data represent mean ± SD; ^∗^*P* < 0.05; ^∗∗^*P* < 0.01. *n* = 3.

**Figure 4:** Autophagy regulated Wnt signaling pathway during hepatic differentiation of HPCs. (a) RT-PCR analyzing the mRNA expression of Wnt1, Wnt3a, Wnt4, Wnt5a, and Wnt9a in WB-F344 cells treated with differentiation medium (HGF) for 2 days and coculture DMSO or rapamycin (200 nM; Rapa) for 24 h. (b) RT-PCR analyzing the mRNA expression of *β*-catenin, Sox9, and Axin2 in WB-F344 cells treated with differentiation medium (HGF) for 2 days and coculture DMSO or rapamycin (200 nM; Rapa) for 24 h. (c) Western blot showing the level of Wnt5a, P-CaMKII*α*, and CaMKII*α* in WB-F344 cells treated with differentiation medium (HGF) for 2 days and coculture DMSO or rapamycin (200 nM; Rapa) for 24 h. (d) Western blot showing the level of Wnt3a, *β*-catenin, and Sox9 in WB-F344 cells treated with differentiation medium (HGF) for 2 days and coculture DMSO or rapamycin (200 nM; Rapa) for 24 h. (e) RT-PCR analyzing the mRNA expression of Wnt1, Wnt3a, Wnt4, Wnt5a, and Wnt9a in WB-F344 cells treated with differentiation medium (HGF) for 2 days and coculture DMSO or starvation (serum-free medium; Starve) for 24 h. (f) RT-PCR analyzing the mRNA expression of *β*-catenin, Sox9, and Axin2 in WB-F344 cells treated with differentiation medium (HGF) for 2 days and coculture DMSO or starvation (serum-free medium; Starve) for 24 h. (g) Western blot showing the level of Wnt5a, P-CaMKII*α*, and CaMKII*α* in WB-F344 cells treated with differentiation medium (HGF) for 2 days and coculture DMSO or starvation (serum-free medium; Starve) for 24 h. (h) Western blot showing the level of Wnt3a, *β*-catenin, and Sox9 in WB-F344 cells treated with differentiation medium (HGF) for 2 days and coculture DMSO or starvation (serum-free medium; Starve) for 24 h. Data represent mean ± SD; ^∗^*P* < 0.05; ^∗∗^*P* < 0.01. *n* = 3.

The article "Autophagy Is Required for Hepatic Differentiation of Hepatic Progenitor Cells via Wnt Signaling Pathway" was published in 2021. Journal: Biomed Res Int.

**Table 1:** Primers used for RT-PCR.

Gene	Sequence (5′-3′)	Product length (bp)
Alb	F: AGAACCAGGCCACTATCTC	110
	R: CAGATCGGCAGGAATGTTGT	
Aldob	F: CTGTGCCTCTTCTCTAACCAAC	152
	R: GAACATCCATCCAAGAGAAGAA	
Wnt1	F: ATGAACCTTCACAATAACGAG	202
	R: GGTTGTTGCCTCGGTTG	
Wnt3a	F: ATTGAATTTGGAGGAATGGT	318
	R: CTTGAAGTATGTGTAACGTG	
Wnt4	F: GAGCAGGACATCCGCAGT	120
	R: CTCCACTTGCGCTGTGTG	
Wnt5a	F: CCAAGTCCGGACTACTGTGT	189
	R: CTTGACATAGCAGCACCAGTG	
Wnt9a	F: ACACTGGTGGAGGCCGTA	151
	R: TCCTTGAAGCCTCGCTTG	
*β*-Catenin	F: AAGTTCTTGGCTATTACGACA	169
	R: ACAGCACCTTCAGCACTCT	
Sox9	F: GAGCCGGATCTGAAGAAGGA	151
	R: GCTTGACGTGTGGCTTGTTC	
Axin2	F: TGACTCTCCTTCCAGATCCAA	105
	R: TGCCCACGCTAGGCTGACA	
Gapdh	F: CCGTGTTCCTACCCCCAATG	116
	R: CCTTTAGTGGGCCCTCGGC	

## Data Availability

The datasets used and/or analyzed during the current study are available from the corresponding author on reasonable request.

## Abbreviations

HPCs: Hepatic progenitor cells
BMP: Bone morphogenetic protein
HGF: Hepatocyte growth factor
FGF: Fibroblast growth factor
ALB: Albumin
Rapa: Rapamycin
Starve: Starvation
RT-PCR: Real-time polymerase chain reaction
CCK8: Cell Counting Kit-8
SD: Standard deviation
DR: Ductular reactions
CaMKII: Calcium/calmodulin-dependent kinase II
GAPDH: Glyceraldehydes-3-phosphate dehydrogenase.

## References

[1] Moon A. M., Singal A. G., Tapper E. B. (2020). Contemporary epidemiology of chronic liver disease and cirrhosis. *Clinical Gastroenterology and Hepatology*.

[2] Yang L. S., Shan L. L., Saxena A., Morris D. L. (2014). Liver transplantation: a systematic review of long-term quality of life. *Liver International*.

[3] Forbes S. J., Newsome P. N. (2016). Liver regeneration - mechanisms and models to clinical application. *Nature Reviews. Gastroenterology & Hepatology*.

[4] Bria A., Marda J., Zhou J. (2017). Hepatic progenitor cell activation in liver repair. *Liver Res*.

[5] Miyajima A., Tanaka M., Itoh T. (2014). Stem/progenitor cells in liver development, homeostasis, regeneration, and reprogramming. *Cell Stem Cell*.

[6] Chen J., Chen L., Zern M. A. (2017). The diversity and plasticity of adult hepatic progenitor cells and their niche. *Liver International*.

[7] Yamashita T., Wang X. W. (2013). Cancer stem cells in the development of liver cancer. *The Journal of Clinical Investigation*.

The article "Autophagy Is Required for Hepatic Differentiation of Hepatic Progenitor Cells via Wnt Signaling Pathway" was published in 2021. Journal: Biomed Res Int.

[8] Michalopoulos G. K., Khan Z. (2015). Liver stem cells: experimental findings and implications for human liver disease. *Gastroenterology*.

[9] Van Camp J. K., Beckers S., Zegers D., Van Hul W. (2014). Wnt signaling and the control of human stem cell fate. *Stem Cell Reviews and Reports*.

[10] van Amerongen R., Nusse R. (2009). Towards an integrated view of Wnt signaling in development. *Development*.

[11] Katoh M. (2017). Canonical and non-canonical WNT signaling in cancer stem cells and their niches: cellular heterogeneity, omics reprogramming, targeted therapy and tumor plasticity (review). *International Journal of Oncology*.

[12] Katoh M., Katoh M. (2007). WNT signaling pathway and stem cell signaling network. *Clinical Cancer Research*.

[13] Clevers H. (2006). Wnt/beta-catenin signaling in development and disease. *Cell*.

[14] Baron R., Kneissel M. (2013). WNT signaling in bone homeostasis and disease: from human mutations to treatments. *Nature Medicine*.

[15] Chavali M., Klingener M., Kokkosis A. G. (2018). Non-canonical Wnt signaling regulates neural stem cell quiescence during homeostasis and after demyelination. *Nature Communications*.

[16] Fan J., Wei Q., Liao J. (2017). Noncanonical Wnt signaling plays an important role in modulating canonical Wnt-regulated stemness, proliferation and terminal differentiation of hepatic progenitors. *Oncotarget*.

[17] Choi A. M. K., Ryter S. W., Levine B. (2013). Autophagy in human health and disease. *The New England Journal of Medicine*.

[18] Mizushima N. (2018). A brief history of autophagy from cell biology to physiology and disease. *Nature Cell Biology*.

[19] Ueno T., Komatsu M. (2017). Autophagy in the liver: functions in health and disease. *Nature Reviews. Gastroenterology & Hepatology*.

[20] Pan H., Cai N., Li M., Liu G. H., Izpisua Belmonte J. C. (2013). Autophagic control of cell ‘stemness’. *EMBO Molecular Medicine*.

[21] Boya P., Codogno P., Rodriguez-Muela N. (2018). Autophagy in stem cells: repair, remodelling and metabolic reprogramming. *Development*.

[22] Lei Y., Zhang D., Yu J., Dong H., Zhang J., Yang S. (2017). Targeting autophagy in cancer stem cells as an anticancer therapy. *Cancer Letters*.

[23] Ho T. T., Warr M. R., Adelman E. R. (2017). Autophagy maintains the metabolism and function of young and old stem cells. *Nature*.

[24] Zeng J., Jing Y., Shi R. (2016). Autophagy regulates biliary differentiation of hepatic progenitor cells through Notch1 signaling pathway. *Cell Cycle*.

[25] Gao C., Cao W., Bao L. (2010). Autophagy negatively regulates Wnt signalling by promoting Dishevelled degradation. *Nature Cell Biology*.

The article "Autophagy Is Required for Hepatic Differentiation of Hepatic Progenitor Cells via Wnt Signaling Pathway" was published in 2021. Journal: Biomed Res Int.

[26] Petherick K. J., Williams A. C., Lane J. D. (2013). Autolysosomal *β*-catenin degradation regulates Wnt-autophagy-p62 crosstalk. *The EMBO Journal*.

[27] Jia Z., Wang J., Wang W. (2014). Autophagy eliminates cytoplasmic *β*-catenin and NICD to promote the cardiac differentiation of P19CL6 cells. *Cellular Signalling*.

[28] Fausto N. (2004). Liver regeneration and repair: hepatocytes, progenitor cells, and stem cells. *Hepatology*.

[29] Williams M. J., Clouston A. D., Forbes S. J. (2014). Links between hepatic fibrosis, ductular reaction, and progenitor cell expansion. *Gastroenterology*.

[30] Clouston A. D., Powell E. E., Walsh M. J., Richardson M. M., Demetris A. J., Jonsson J. R. (2005). Fibrosis correlates with a ductular reaction in hepatitis C: roles of impaired replication, progenitor cells and steatosis. *Hepatology*.

[31] Roskams T. A., Theise N. D., Balabaud C. (2004). Nomenclature of the finer branches of the biliary tree: canals, ductules, and ductular reactions in human livers. *Hepatology*.

[32] Gordon M. D., Nusse R. (2006). Wnt signaling: multiple pathways, multiple receptors, and multiple transcription factors. *The Journal of Biological Chemistry*.

[33] Mikels A. J., Nusse R. (2006). Purified Wnt5a protein activates or inhibits beta-catenin-TCF signaling depending on receptor context. *PLoS Biology*.

[34] Liang H., Chen Q., Coles A. H. (2003). Wnt5a inhibits B cell proliferation and functions as a tumor suppressor in hematopoietic tissue. *Cancer Cell*.

[35] Guan J. L., Simon A. K., Prescott M. (2013). Autophagy in stem cells. *Autophagy*.

[36] Cheng Y., Wang B., Zhou H. (2015). Autophagy is required for the maintenance of liver progenitor cell functionality. *Cellular Physiology and Biochemistry*.

[37] Ren L., Han W., Yang H. (2016). Autophagy stimulated proliferation of porcine PSCs might be regulated by the canonical Wnt signaling pathway. *Biochemical and Biophysical Research Communications*.

